The article "Application of Deep Neural Network Model Combined with Factor Analysis in Clinical Nursing Effect Analysis of Blood Glucose Level in Elderly Type 2 Diabetic Patients" was retracted in 2023. Reason: concerns about the peer review.

# Application of Deep Neural Network Model Combined with Factor Analysis in Clinical Nursing Effect Analysis of Blood Glucose Level in Elderly Type 2 Diabetic Patients

**DOI:** 10.1155/2021/3462128

**Published:** 2021-09-13

**Authors:** Yi Ding, DanDan Zhang

**Affiliations:** Department of Endocrinology, Tangshan Central Hospital, Hebei 063000, China

## Abstract

In order to explore the clinical nursing effect of blood glucose level in elderly type 2 diabetic patients, this paper combines the deep neural network model and factor analysis from the perspective of multifactor analysis to construct a multifactor analysis model for the clinical nursing effect of blood glucose levels in elderly type 2 diabetic patients. Moreover, this paper analyzes the effects through experimental methods, collects cases through hospitals, and formulates research methods and related standards based on nursing research needs. In addition, this paper uses statistical methods to perform data processing, uses factor analysis to screen critical factors, and uses deep neural networks to process nursing data. The statistical results of the experimental research show that the deep neural network model combined with factor analysis can play a certain role in the clinical nursing effect. Thus, the blood glucose level analysis in elderly type 2 diabetic patients can provide a reference direction for the clinical care of blood glucose levels in elderly type 2 diabetic patients.

## 1. Introduction

The physiology of elderly type 2 diabetes patients is quite special. With the increase of age, the incidence rate gradually increases. Meanwhile, the patient has the following characteristics: (1) The patient's condition is hidden and often serious, and the early symptoms of the patient are not typical, which is easily missed and misdiagnosed [1]. (2) Patients often have many kinds of diseases from other systems, and cardiovascular diseases are most often involved. (3) The ability to resist various infections decreases often leads to infections in various parts and further increases the difficulty of controlling blood sugar to reach the standard. (4) The patient's psychological factors easily affect the condition [2]. (5) Due to the complex condition of the disease, it is necessary to cross-administer drugs with different diseases, which leads to a decline in the patient's metabolic capacity and limits the use of hypoglycemic drugs. (6) Patients often cannot take care of themselves independently, have poor memory ability, and cannot take hypoglycemic drugs on time, which indirectly affects the control of blood sugar levels [3]. HbA1c is produced by the reaction between hemoglobin and blood sugar in the human body, and it increases with the increase of blood sugar concentration. It can indirectly show blood glucose changes in the patient's body in the last 8–12 weeks and has become a leading indicator used to monitor whether the patient's blood glucose control meets the standard [4]. The blood sugar control of diabetic patients is affected by many factors, such as whether the corresponding diet and exercise treatment plan given by the doctor is appropriate, whether the patient can implement it according to the plan, and the strength of the implementation. Secondly, if the patient has serious cardiopulmonary disease, bone and joint disease, etc., it will also affect their blood sugar control. In addition, the type and quantity of drugs taken by patients, whether they can take them on time, the number of insulin treatments, and the amount of each application are all factors that affect blood sugar control [5].

The article "Application of Deep Neural Network Model Combined with Factor Analysis in Clinical Nursing Effect Analysis of Blood Glucose Level in Elderly Type 2 Diabetic Patients" was retracted in 2023. Reason: concerns about the peer review.

This article analyzes the impact of health education on the level of blood glucose control in elderly type 2 diabetic patients.

## 2. Related Work

The bone tissue morphology of diabetic animal models provides evidence for the study of bone mineralization and bone transformation rate. Through the morphological examination of diabetic rats, the literature [6] found that the markers of osteoblasts including osteoid thickness, osteoid surface area, and osteoid volume significantly reduced. Furthermore, bone tissue dynamic parameters such as bone mineralization surface area were significantly reduced. In addition, osteoclast-marked bone erosion surface significantly increased, which indicated that the osteoblast activity of diabetic rats decreases, bone formation decreases, and bone resorption increases. In terms of biomechanics, the three-point bending test showed that the femur's maximum load, stiffness, and energy absorption were significantly reduced, indicating an increase in bone fragility. On the other hand, the elastic modulus of the femur did not change substantially in the lumbar spine compression test. Still, the lumbar spine's elastic modulus and maximum load did, suggesting that the lumbar spine rich in cancellous bone may be more vulnerable to diabetes than the femur.

One of the reasons for the increase of bone fragility in diabetic patients is the increase in the concentration of advanced glycation end products (AGE) of bone collagen, which leads to changes in the physical and chemical properties of the collagen matrix. The effect of AGE on osteoblasts has been studied in depth. Integrins play a role in adhering cells and collagen as a receptor for osteoblasts on the surface of type I collagen. The literature [7] synthesized integrin subunits located on collagen to recognize peptide chains RGD and DGEA. These exogenous peptide chains competitively inhibited the connection between osteoblasts and collagen but did not significantly inhibit the connection between osteoblasts and AGE-modified collagen. Thus, it shows that AGE-modified type I collagen destroys integrin-mediated adhesion of osteoblasts and collagen. The literature [8] isolated fetal rat skull osteoblasts and cultured in AGE-modified type I collagen. The results show an inhibitory effect on AGE concentration-dependent osteoblast characteristics. Moreover, the results show that the formation of bone nodules was inhibited by 70% at 1 week, and bone alkaline phosphatase and osteocalcin were also inhibited to a certain extent at 5 weeks. The above results indicate that in vitro AGE-modified collagen inhibits the differentiation and function of osteoblasts. However, when the literature [9] studied the effect of AGE on the differentiation of human bone marrow mesenchymal stem cells, it was found that after 3 weeks AGE increased bone alkaline phosphatase activity and intracellular calcium concentration, but the formation of mineralized nodules was inhibited. The reason for the difference in the above research results is not clear. It may be related to the measurement time of the index and the degree of cell differentiation. However, AGE certainly has an inhibitory trend in the overall function of osteoblasts.

The article "Application of Deep Neural Network Model Combined with Factor Analysis in Clinical Nursing Effect Analysis of Blood Glucose Level in Elderly Type 2 Diabetic Patients" was retracted in 2023. Reason: concerns about the peer review.

Many people with type 2 diabetes are overweight or obese. This increase in weight compared to people of the same age adds mechanical stress to the bones, which is equivalent to continuous weight-bearing training for the bones, and repeated mechanical stress stimulation will inevitably lead to an increase in bone density [10]. Adipocytes also release leptin, which may operate directly on bone marrow stromal cells to increase osteoblast development and bone matrix mineralization and encourage osteoblasts to generate osteoprotectin, encouraging bone formation [11]. However, investigations in mice have demonstrated that leptin produced by adipocytes may decrease bone formation by stimulating the 2-adrenergic response system through the leptin receptor in the hypothalamus [12]. Adipocytes may also produce adiponectin, which promotes osteoblast development while inhibiting osteoclast formation [13].

In addition, obesity is associated with type 2 diabetes. In the past, obesity was considered to be a bone protective factor, but recent studies have found that obesity can cause more bone damage [14]. Moreover, obesity can activate the nuclear receptor peroxisome proliferator-activated receptor *γ* (PPAR*γ*), which is an important factor in adipocyte differentiation. It can promote the differentiation of stromal stem cells in bone marrow to adipocytes but not osteoblasts and inhibit the differentiation and function of osteoblasts. Furthermore, obesity can aggravate oxidative stress and release inflammatory factors such as tumor necrosis factor-alpha and interleukin 1-beta.

The article "Application of Deep Neural Network Model Combined with Factor Analysis in Clinical Nursing Effect Analysis of Blood Glucose Level in Elderly Type 2 Diabetic Patients" was retracted in 2023. Reason: concerns about the peer review.

On the one hand, these inflammatory factors stimulate the formation of mononuclear macrophages and transform into osteoclasts, strengthen the activity of osteoclasts and bone resorption, and on the other hand promote the apoptosis of osteoblasts. Inflammatory factors can also promote the expression and secretion of RANKL (receptor activator of nuclear factor-*κ*B ligand) by osteoblasts. The latter is the most important factor that promotes osteoclasts' differentiation, maturation, and functional activity. Therefore, obesity affects the bone remodeling process through different mechanisms, and the role of bone damage may be dominant [15].

Diabetic neuropathy is the most common chronic complication of diabetes. The relationship between neuropathy and falls in diabetic patients has attracted widespread attention. The literature [16] found that women with diabetes who had a fall in the past year had a higher vibration threshold, but no relationship between the 10 g nylon tactile test results and the fall was found. The reason may be that this test is not sensitive to patients with early sensory nerve function impairment. Another prospective study [17] showed that patients who fell more than once a year had decreased shock sensitivity and pressure sensitivity. The OR after adjusting for age were 1.12 (95% CI: 1.05–1.19) and 1.58 (95% CI: 1.34–1.87), respectively. Moreover, neurological complications may affect the patient's gait, walking speed, and balance ability [18], and the slowing of nerve conduction velocity may also be one of the risk factors for falls [19]. However, some studies [20] did not find a significant correlation between neuropathy and falls.

## 3. Boltzmann Machine Network and RBM Network

The Boltzmann Machine algorithm (Boltzmann Machine, BM) was proposed by researchers as early as the 1980s. It is a probabilistic graph model composed of visible layers and hidden layers and can learn the dependencies between visible layer units.

As shown in Figure 1(a), the BM model consists of a set of visible layer unit,

(1) $$\begin{array}{c} v={\left\{v_{i}\right\}}_{i=1}^{D}, \end{array}$$

and hidden layer unit,

(2) $$\begin{array}{c} h={\left\{h_{i}\right\}}_{i=1}^{J}. \end{array}$$

At this time, the energy function and likelihood function of BM can be expressed as

(3) $$\begin{array}{c} E\left(v,h;\theta \right)=-\overset{D}{\underset{i=1}{\sum }}\overset{J}{\underset{j=1}{\sum }}v_{i}W_{ij}h_{j}-\frac{1}{2}\overset{D}{\underset{i=1}{\sum }}\overset{D}{\underset{i^{\prime }=1}{\sum }}v_{i}L_{ii{}^{\prime }}v_{i^{\prime }}\\ -\frac{1}{2}\sum_{j=1}^{J}\overset{J}{\underset{j^{\prime }=1}{\sum }}h_{j}M_{jj^{\prime }}h_{j^{\prime }}-\overset{D}{\underset{i=1}{\sum }}C_{i}v_{i}-\sum_{j=1}^{J}b_{j}h_{j},\\ P\left(v;\theta \right)=\underset{h}{\sum }P\left(v,h;\theta \right)=\frac{1}{Z\left(\theta \right)}\underset{h}{\sum }\exp\left(-E\left(v,h;\theta \right)\right). \end{array}$$

Among them,

(4) $$\begin{array}{c} \theta =\left\{W,WL,M,c,b\right\}, \end{array}$$

is the network weight in the BM model. *W* represents the connection weight between the visible and hidden layers, *L* and *M*, respectively, represent the connection weight between the visible and hidden layers, and *c* and *b*, respectively, represent the bias on the visible and hidden layers.

(5) $$\begin{array}{c} Z\left(\theta \right)=\sum {}_{v}\sum {}_{h}\exp\left(-E\left(v,h;\theta \right)\right), \end{array}$$

is the partition function of BM. Moreover, since LM represents the connection weight inside the visible or hidden layers, the diagonal elements of LM are set to zero. When the states of the visible layer and the hidden layer in the model are fixed, the conditional probability distribution of a certain visible layer unit or a certain hidden layer unit in BM can be calculated:

(6) $$\begin{array}{c} P\left(v_{i}=1|h\right)=\sigma \left(\sum {}_{j}W_{ij}h_{j}+\sum {}_{k\neq i}L_{ik}V_{k}+c_{i}\right),\\ P\left(h_{j}=1|v\right)=\sigma \left(\sum {}_{i}v_{i}W_{ij}+\sum {}_{k\neq j}M_{jk}h_{k}+b_{j}\right). \end{array}$$

Among them,

(7) $$\begin{array}{c} \sigma \left(x\right)=\frac{1}{\left(1+\exp\left(-x\right)\right)}, \end{array}$$

where *b* represents the Sigmoid activation function. The BM model obtains the parameters of the model by maximizing the likelihood function training; and the gradient of the weight can be expressed as the difference between the data-related statistics and the model-related statistics.

(8) $$\begin{array}{c} \Delta W=\alpha \left(E_{P_{data}}\left[vh^{T}\right]-E_{P_{\mathrm{mod}el}}\left[vh^{T}\right]\right),\\ \Delta L=\alpha \left(E_{P_{data}}\left[vv^{T}\right]-E_{P_{\mathrm{mod}el}}\left[vv^{T}\right]\right),\\ \Delta M=\alpha \left(E_{P_{data}}\left[hh^{T}\right]-E_{P_{\mathrm{mod}el}}\left[hh^{T}\right]\right),\\ \Delta c=\alpha \left(E_{P_{data}}\left[v\right]-E_{P_{\mathrm{mod}el}}\left[v\right]\right),\\ \Delta b=\alpha \left(E_{P_{data}}\left[h\right]-E_{P_{\mathrm{mod}el}}\left[h\right]\right). \end{array}$$

Among them, *α* represents the learning rate, *E*_*P*_*data*__[·] represents data-related statistics, and *E*_*P*_mod*el*__[·] represents model-related statistics.

The article "Application of Deep Neural Network Model Combined with Factor Analysis in Clinical Nursing Effect Analysis of Blood Glucose Level in Elderly Type 2 Diabetic Patients" was retracted in 2023. Reason: concerns about the peer review.

In fact, the partition function of BM is difficult to calculate, and the accurate calculation of the maximum likelihood function is very difficult to handle. The computational complexity of BM's data-related statistics is exponential with the number of hidden layer units. At the same time, the calculation complexity of BM's model data-related statistics and the sum of the number of visible layer and hidden layer units are also exponential.

As shown in Figure 1, Restricted Boltzmann Machine (RBM) limits the intralayer connections of BM. As shown in Figure 1(b), if the RBM model is also composed of a set of visible layer units *v*={*v*_*i*_}_*i*=1_^*D*^ and hidden layer units *h*={*h*_*i*_}_*i*=1_^*J*^, then the energy function of RBM can be expressed as

(9) $$\begin{array}{c} E\left(v,h;\theta \right)=-\sum_{i=1}^{D}\sum_{j=1}^{J}v_{i}W_{ij}h_{j}-\sum_{i=1}^{D}C_{i}v_{i}-\sum_{j=1}^{J}b_{j}h_{j}. \end{array}$$

Here, *θ*={*W*, *c*, *b*} is the network weight in the RBM model. When any of the visible layer and the hidden layer in the RBM is in a fixed state, the conditional probability distribution of the other layer can be calculated:

(10) $$\begin{array}{c} P\left(v_{i}=1|h\right)=\sigma \left(\sum {}_{j}W_{ij}h_{j}+c_{i}\right),\\ P\left(h_{j}=1|v\right)=\sigma \left(\sum {}_{i}v_{i}W_{ij}+b_{j}\right). \end{array}$$

Like BM, RBM maximizes the likelihood function training to obtain the parameters of the model. However, since RBM restricts the intralayer connections of BM, the accurate calculation of the RBM maximization likelihood function is much simpler than that of the BM model. In this way, the calculation of RBM data-related statistics can be obtained through variational inference. The lower bound of the log-likelihood function of RBM can be expressed as

(11) $$\begin{array}{c} InP_{\theta }\left(v\right)=In\sum_{h}P_{\theta }\left(v,h\right)=In\sum_{h}Q_{\mu }\left(h|v\right)\cdot \frac{P_{\theta }\left(v,h\right)}{Q_{\mu }\left(h|v\right)}\\ \geq \sum_{h}Q_{\mu }\left(h|v\right)In\left(\frac{P_{\theta }\left(v,h\right)}{Q_{\mu }\left(h|v\right)}\right)\\ =E_{Q_{\mu }\left(h|v\right)}\left[InP_{\theta }\left(v,h\right)\right]-KL\left[Q_{\mu }\left(h|v\right)\left\|P_{\theta }\left(v,h\right)\right.\right]\\ =L\left(Q,\theta \right). \end{array}$$

Here, *Q*_*μ*_(*h|v*) is an approximate posterior of the actual posterior *P*_*θ*_(*v*, *h*), and *L*(*Q*, *θ*) is the lower bound of the log-likelihood function. In order to eliminate the phenomenon of explanation and elimination, the uniform field approximation method is used to approximate the actual posterior *P*_*θ*_(*v*, *h*).

(12) $$\begin{array}{c} Q\left(h;\mu \right)=\prod {}_{j=1}^{j}q\left(h_{j}\right),\\ q\left(h_{j}=1\right)=\mu_{j}. \end{array}$$

Then, *L*(*Q*, *θ*) is expressed as

(13) $$\begin{array}{c} L\left(Q,\theta \right)=\sum_{i=1}^{D}\sum_{j=1}^{J}v_{i}W_{ij}\mu_{j}+\sum_{j=1}^{J}b_{j}\mu_{j}+\sum_{i=1}^{D}C_{i}v_{i}\\ -InZ\left(\theta \right)-\sum_{j=1}^{J}\left(\mu_{j}In\mu_{j}+\left(1-\mu_{j}\right)In\left(1-\mu_{j}\right)\right). \end{array}$$

Therefore, when weight *θ* is fixed and the partial derivative of *L*(*Q*, *θ*) on *μ*_*j*_ is set to zero, we can get

(14) $$\begin{array}{c} \mu_{j}=\sigma \left(\sum {}_{i}v_{i}W_{ij}+b_{j}\right). \end{array}$$

In this way, the hidden layer output obtained by variational inference is consistent with the result obtained by conditional probability sampling.

The article "Application of Deep Neural Network Model Combined with Factor Analysis in Clinical Nursing Effect Analysis of Blood Glucose Level in Elderly Type 2 Diabetic Patients" was retracted in 2023. Reason: concerns about the peer review.

At present, the training of RBM networks often encounters overfitting problems. Commonly used solutions include weight attenuation, dropout, DropConnect, and weight uncertainty. The weight decay method is to add regularization during the training of the weight learning in small batches. Taking the calculation of the gradient of weight *W* as an example, the gradient of weight *W* can be expressed as

(15) $$\begin{array}{c} \Delta W=\alpha \left(E_{P_{data}}\left[vh^{T}\right]-E_{P_{\mathrm{mod}el}}\left[vh^{T}\right]\right)+momentum\times \Delta W^{\prime }. \end{array}$$

Here, momentum represents the weight attenuation coefficient, and Δ*W*′ represents the gradient learned from the previous mini-batch block.

In Dropout RBM (DRBM), the output of the hidden layer is related to a set of binary variables *r*={0,1}^*j*^. If the value of *r*_*j*_ is equal to 1, the corresponding hidden layer output remains unchanged; otherwise it is 0. The probability that the value of *r*_*j*_ is equal to 1 is *p*. At this time, the energy function of DRBM can be expressed as

(16) $$\begin{array}{c} E\left(v,h|r;\theta \right)=-\sum_{i=1}^{D}\sum_{j=1}^{J}v_{i}W_{ij}\left(r_{j}h_{j}\right)-\sum_{j=1}^{J}b_{j}\left(r_{j}h_{j}\right)-\sum_{i=1}^{D}C_{i}v_{i}. \end{array}$$

When any of the visible and hidden layers in DRBM is in a fixed state, the conditional probability distribution of the other layer can be calculated:

(17) $$\begin{array}{c} P\left(h_{j}=1|v,r_{j}\right)=r_{j}\cdot \sigma \left(\sum {}_{i}v_{i}W_{ij}+b_{j}\right),\\ P\left(v_{i}=1|h,r\right)=\sigma \left(\sum {}_{j}W_{ij}\left(r_{j}h_{j}\right)+c_{i}\right). \end{array}$$

In DropConnect RBM (DcRBM), the weights connecting visible and hidden units are related to a set of binary matrices *M* ∈ *R*^*D*×*J*^. If the value of *M*_*ij*_ is equal to 1, the corresponding connection weight *W*_*ij*_ remains unchanged; otherwise it is 0. Moreover, the probability that the value of *M*_*ij*_ is equal to 1 is *p*. At this time, the energy function of DcRBM can be expressed as

(18) $$\begin{array}{c} E\left(v,h|M;\theta \right)=-\sum_{i=1}^{D}\sum_{j=1}^{J}v_{i}\left(\frac{W_{ij}M_{ij}}{P}\right)h_{j}-\sum_{j=1}^{J}b_{j}h_{j}-\sum_{i=1}^{D}C_{i}v_{i}. \end{array}$$

When any of the visible and hidden layers in DcRBM is in a fixed state, the conditional probability distribution of the other layer can be calculated:

(19) $$\begin{array}{c} P\left(h_{j}=1|v,M\right)=\sigma \left(\sum_{i}v_{i}\left(\frac{W_{ij}M_{ij}}{P}\right)+b_{j}\right),\\ P\left(v_{i}=1|h,M\right)=\sigma \left(\sum_{j}\left(\frac{W_{ij}M_{ij}}{P}\right)h_{j}+c_{i}\right). \end{array}$$

The article "Application of Deep Neural Network Model Combined with Factor Analysis in Clinical Nursing Effect Analysis of Blood Glucose Level in Elderly Type 2 Diabetic Patients" was retracted in 2023. Reason: concerns about the peer review.

## 4. Research Methods

This article uses deep neural network model combined with factor analysis to analyze the clinical nursing effect of blood glucose levels in elderly type 2 diabetic patients.

In the experiment, 114 elderly patients with type 2 diabetes and cataract surgery from January 2019 to December 2020 were selected and divided into two groups by the random number table, 57 cases in each group. Among them, there were 28 females and 27 males in the study group: ages of 61–78 (69.13 ± 4.21) years with 21 cases of left eye disease and 21 cases of right eye disease. In the control group, there were 26 females and 29 males: ages of 63–76 (68.89 ± 4.27) years with 20 cases of left eye disease and 22 cases of right eye disease. There was no statistically significant difference between the two groups of general information (*p* > 0.05), and they were comparable. The Medical Ethics Committee approved the study.

In the experiment, the blood glucose control of patients was divided into the three following groups based on HbA1c level: Group I: good blood sugar control, HbA1c < 7.0%; Group II: normal blood sugar control, 7.0 ≤ HbA1c < 9.0%; and Group III: poor blood sugar control, HbA1c ≥ 9.0%.

Methods of controlling blood sugar include diet control, exercise, oral hypoglycemic drugs, or insulin therapy. Exclusion criteria were as follows: (1) type 1 diabetes, (2) acute and chronic infectious diseases, (3) drug exocrine pancreatic diseases, (4) endocrine diseases such as hypercortisolism, (5) patients with severe mental and/or neurological diseases, (6) patients with chronic liver and kidney diseases, (7) patients treated with glucocorticoids, (8) patients with anemia and hematological diseases, (9) patients with a history of drug or alcohol dependence, (10) patients with autoimmune diseases, and (11) patients who use drugs that affect the immune response.

The article "Application of Deep Neural Network Model Combined with Factor Analysis in Clinical Nursing Effect Analysis of Blood Glucose Level in Elderly Type 2 Diabetic Patients" was retracted in 2023. Reason: concerns about the peer review.

Before the experiment, it is essential to inquire for medical history and record basic information, including age, course of DM, altitude of habitual habitation, complications and severity of DM, prevalence of cardiovascular and respiratory illnesses, and cerebrovascular diseases. All participants' height (BH), weight, waist circumference (WC), systolic blood pressure (SBP), diastolic blood pressure (DBP), and body mass index (BMI) were taken after they awoke on an empty stomach (fasting for more than 8 hours).

In the experiment, 10 ml of cubital venous blood was collected and submitted for examination. A part was used to measure glycosylated hemoglobin (HbA1c), fasting blood glucose (FBG), and postprandial blood glucose (PBG). The other part was used to determine biochemical indicators (TG, TCH, HDL-C, LDL-C, HGB, RBC, and MCV). After the collected data were comprehensive, statistical analysis will be performed. The grading standard of DM complications and severity refers to the grading standard of scientific research methods of metabolic syndrome commonly used in the endocrine system. Furthermore, the experiment was graded based on the existence of metabolic syndrome in each system component, with each syndrome receiving one point. Cardiovascular illnesses like premature atrial flutter, ventricular flutter, pericardial effusion, aortic valve calcification, tricuspid valve regurgitation, aortic valve calcification and regurgitation, and pulmonary valve regurgitation were all mentioned.

Respiratory diseases such as chronic bronchitis, emphysema, pulmonary hypertension, lung inflammation, pleural effusion, interstitial pulmonary fibrosis, pulmonary heart disease, and respiratory failure were also scored according to the number of diseases. In addition, cerebrovascular diseases such as cerebral infarction, cerebral ischemia, senile brain, and other diseases were scored by the number of diseases. According to the above method, the prevalence of cardiovascular and respiratory diseases and cerebrovascular diseases was converted into scores and quantified as observation indicators. The scores of different system diseases were accumulated in sequence and analyzed statistically.

In the statistical method, the experiment uses SPSS 19.0 statistical software to analyze the data, and the measurement data results are expressed as mean ± standard deviation (*x* ± *S*). Moreover, the significance test between the groups uses one-way analysis of variance, the pairwise comparison uses the LSD test method, and the regression analysis is performed simultaneously. Finally, the count data uses the *χ*^2^ test, and the test level is *α* = 0.05.

The article "Application of Deep Neural Network Model Combined with Factor Analysis in Clinical Nursing Effect Analysis of Blood Glucose Level in Elderly Type 2 Diabetic Patients" was retracted in 2023. Reason: concerns about the peer review.

This article analyzes the influencing factors through experimental research, including age, course of DM, complications of DM, cardiopulmonary disease, cerebrovascular disease, permanent low altitude, and other factors. Moreover, this paper uses factor analysis to obtain the above-mentioned main factors, analyzes these influencing factors through the deep neural network model of this paper, and develops targeted nursing methods. In addition, this paper uses the sample data of this paper as input and uses deep neural network to process the data and get the corresponding results.

First, this paper analyzes the correlation between age and the clinical nursing effect of blood glucose levels in elderly type 2 diabetic patients, and the results are shown in Figure 2 and Table 1.

This article analyzes the correlation between the course of DM and the clinical nursing effect of blood glucose levels in elderly type 2 diabetic patients, and the results are shown in Figure 3 and Table 2.

This article analyzes the correlation between the DM complications and the clinical nursing effect of blood glucose levels in elderly type 2 diabetic patients, and the results are shown in Figure 4 and Table 3.

This article analyzes the correlation between cardiopulmonary diseases and the clinical nursing effect of blood glucose levels in elderly type 2 diabetic patients, and the results are shown in Figure 5 and Table 4.

Figure 6 and Table 5 demonstrate the results of this study on the relationship between cerebrovascular illnesses and the clinical nursing effect of blood glucose levels in older type 2 diabetic patients.

This article analyzes the correlation between the resident at low altitude and the clinical nursing effect of blood glucose levels in elderly type 2 diabetic patients, and the results are shown in Figure 7 and Table 6.

The pancreatic islet function of the elderly gradually declines with age. As the age continues to increase, INS resistance will gradually increase with the increase of age. Moreover, the body's resistance to the outside world will be low for older people, and infection will occur easily. The condition is easily disturbed by psychological reasons. Moreover, patients often have different systemic diseases and need to cross medication, so hypoglycemic drugs are limited. As a result, patients' blood sugar increases with age and becomes more and more difficult to control. In addition, the cognition level of the elderly gradually decreases with age. The main manifestations are poor ability to accept new things, inability to strictly follow the doctor's instructions for diet and exercise treatment, and inability to use oral medication or insulin on time, and some patients even use the wrong medication, which will affect the patient's blood sugar control.

The article "Application of Deep Neural Network Model Combined with Factor Analysis in Clinical Nursing Effect Analysis of Blood Glucose Level in Elderly Type 2 Diabetic Patients" was retracted in 2023. Reason: concerns about the peer review.

When the patient has pulmonary heart disease, it will cause insulin resistance in the body itself. If the patient is in a more serious condition, the pancreatic islet B cells will be severely damaged, and the body will secrete more hormones that raise blood sugar than usual. Moreover, the liver's glucose metabolism is lower than normal. All of the above factors make it difficult to control blood sugar. In patients with coronary heart disease, because they cannot eat foods high in sodium or fat, they will gradually change their diet and eat some foods with high starch and high sugar content.

Moreover, the patient's heart burden is very heavy and they canno't do too much activity, making it difficult to control blood sugar after a meal. Drugs used to treat cardiovascular diseases may also affect glucose metabolism, so blood sugar and HbA1c levels increase. Patients with the cerebrovascular disease will have reduced self-care ability, irregular diet and medication, and restricted exercise after meals, which will cause poor blood sugar control.

With the prolongation of the course of DM, blood sugar will become more and more difficult to control. At this time, B-cell function gradually declines, insulin concentration in the body decreases with the course of the disease, and blood sugar is more difficult to control, which is consistent with this result.

Diabetes itself does not cause serious physical harm to patients. However, long-term hyperglycemia may cause various concurrent diseases, and diabetes can cause great pressure on major body organs such as the heart and brain blood vessels, liver, and kidneys and may be fatal in critical conditions. Patients with diabetic retinopathy have lower self-care ability than normal people, and oral medication and insulin are restricted. The INS of patients with DM nephropathy will slowly accumulate in the human body and cannot be excreted normally. Patients with peripheral neuropathy will have numbness and pain in their limbs, and the patient's mood will be poor, sleep will be affected, and blood sugar will also change accordingly. In addition, patients with acute complications of DM have insufficient secretion of INS, which has a more pronounced impact on HbA1c levels.

Under high altitude stimulation, various metabolic rates in the human body will increase, disturbing the source and the way of glucose and leading to increased blood sugar.

## 5. Conclusion

Elderly type 2 diabetic patients have poor overall blood glucose control, and most patients have high blood glucose levels. In nursing, it is necessary to formulate targeted nursing strategies from age, DM course, complications of DM, cardiopulmonary disease, cerebrovascular disease, permanent low altitude, and other factors. At the same time, it is necessary to strengthen the publicity and education of patients' health and safety knowledge, enhance the awareness of patients, and enable patients to truly realize the role and significance of continuous diet care in diabetic patients. At the same time, it is necessary to pay attention to the psychological counseling of patients so that patients can actively obey nursing work and implement continuous diet care. In addition, it is necessary to provide patients with a scientific diet plan from a health point of view and prohibit patients from eating foods that are not conducive to the recovery of patients and ensure that the food is easy to digest and absorb. Finally, it is necessary to effectively stabilize the patient's blood sugar level and stabilize the patient's condition under diet care and medication intervention.

The article "Application of Deep Neural Network Model Combined with Factor Analysis in Clinical Nursing Effect Analysis of Blood Glucose Level in Elderly Type 2 Diabetic Patients" was retracted in 2023. Reason: concerns about the peer review.

## Figures and Tables

**Figure 1:** Network structure of (a) BM and (b) RBM models.

**Figure 2:** Statistical diagram of the correlation between age and the clinical care effect of blood glucose levels in elderly type 2 diabetic patients.

**Figure 3:** Statistical diagram of the correlation between the course of DM and the clinical nursing effect of blood glucose levels in elderly type 2 diabetic patients.

**Figure 4:** Statistical diagram of the correlation between DM complications and the clinical nursing effect of blood glucose levels in elderly type 2 diabetic patients.

**Figure 5:** Statistical diagram of the correlation between cardiopulmonary diseases and the clinical nursing effect of blood glucose levels in elderly type 2 diabetic patients.

**Figure 6:** Statistical diagram of the correlation between cerebrovascular diseases and the clinical nursing effect of blood glucose levels in elderly type 2 diabetic patients.

**Figure 7:** Statistical diagram of the correlation between the resident at low altitude and the clinical nursing effect of blood glucose levels in elderly type 2 diabetic patients.

**Table 1:** Statistical diagram of the correlation between age and the clinical nursing effect of blood glucose levels in elderly type 2 diabetic patients.

No.	Correlation	No.	Correlation	No.	Correlation
1	95.3	13	93.5	25	92.4
2	96.0	14	93.7	26	90.7
3	93.8	15	96.3	27	94.8
4	88.9	16	93.6	28	95.3
5	91.2	17	91.9	29	95.2
6	93.7	18	94.4	30	94.8
7	89.2	19	89.9	31	92.7
8	93.2	20	93.4	32	89.4
9	88.4	21	88.2	33	96.4
10	90.2	22	95.8	34	95.8
11	91.2	23	90.6	35	95.1
12	89.9	24	95.6		

**Table 2:** Statistical table of the correlation between the course of DM and the clinical nursing effect of blood glucose levels in elderly type 2 diabetic patients.

No.	Correlation	No.	Correlation	No.	Correlation
1	82.5	13	84.8	25	90.5
2	82.9	14	80.8	26	89.4
3	84.4	15	87.8	27	83.1
4	87.9	16	91.9	28	81.2
5	85.7	17	83.6	29	91.2
6	86.3	18	90.2	30	91.7
7	88.5	19	81.3	31	88.5
8	87.7	20	83.3	32	84.2
9	86.2	21	91.9	33	90.1
10	87.6	22	83.8	34	90.6
11	83.6	23	80.3	35	83.1
12	84.6	24	85.5		

The article "Application of Deep Neural Network Model Combined with Factor Analysis in Clinical Nursing Effect Analysis of Blood Glucose Level in Elderly Type 2 Diabetic Patients" was retracted in 2023. Reason: concerns about the peer review.

**Table 3:** Statistical table of the correlation between DM complications and the clinical nursing effect of blood glucose levels in elderly type 2 diabetic patients.

No.	Correlation	No.	Correlation	No.	Correlation
1	93.2	13	91.0	25	90.2
2	84.9	14	87.0	26	85.1
3	90.0	15	88.3	27	87.2
4	92.4	16	86.7	28	85.5
5	93.5	17	88.9	29	87.9
6	89.2	18	91.1	30	92.3
7	88.9	19	93.9	31	86.5
8	86.6	20	93.8	32	91.5
9	87.4	21	91.6	33	85.0
10	85.2	22	84.2	34	87.2
11	93.0	23	89.8	35	91.8
12	91.7	24	90.3		

**Table 4:** Statistical table of the correlation between cardiopulmonary diseases and the clinical nursing effect of blood glucose levels in elderly type 2 diabetic patients.

No.	Correlation	No.	Correlation	No.	Correlation
1	82.7	13	90.5	25	82.5
2	82.8	14	79.6	26	88.9
3	83.5	15	90.8	27	81.2
4	89.2	16	91.4	28	87.3
5	81.4	17	82.8	29	88.1
6	89.0	18	84.2	30	84.7
7	82.4	19	87.3	31	90.3
8	80.2	20	81.4	32	90.2
9	83.4	21	87.2	33	91.6
10	82.9	22	82.1	34	82.7
11	83.9	23	88.2	35	79.0
12	83.6	24	82.8		

**Table 5:** Statistical table of the correlation between cerebrovascular diseases and the clinical nursing effect of blood glucose levels in elderly type 2 diabetic patients.

No.	Correlation	No.	Correlation	No.	Correlation
1	81.5	13	81.8	25	92.3
2	88.9	14	88.8	26	92.0
3	80.8	15	88.4	27	81.4
4	84.8	16	92.3	28	87.3
5	90.7	17	87.4	29	84.4
6	80.1	18	89.2	30	85.7
7	81.2	19	90.0	31	87.2
8	83.1	20	85.4	32	91.2
9	86.7	21	86.7	33	81.7
10	92.0	22	84.8	34	92.2
11	92.4	23	91.7	35	86.9
12	87.4	24	87.7		

**Table 6:** Statistical table of the correlation between the resident at low altitude and the clinical nursing effect of blood glucose levels in elderly type 2 diabetic patients.

No.	Correlation	No.	Correlation	No.	Correlation
1	81.8	13	85.1	25	87.5
2	81.1	14	83.7	26	86.4
3	82.3	15	81.5	27	88.0
4	84.4	16	86.8	28	83.1
5	81.8	17	83.0	29	82.1
6	87.1	18	82.2	30	85.6
7	84.0	19	85.9	31	81.4
8	81.9	20	85.9	32	83.3
9	81.2	21	87.8	33	83.9
10	85.0	22	82.8	34	83.3
11	86.4	23	86.9	35	81.4
12	82.8	24	84.5		

## Data Availability

The data used to support the findings of this study are included within the article.
